# MiR-365a-3p-Mediated Regulation of HELLS/GLUT1 Axis Suppresses Aerobic Glycolysis and Gastric Cancer Growth

This article has been retracted.

**DOI:** 10.3389/fonc.2021.616390

**Published:** 2021-03-15

**Authors:** Rui Yang, Gen Liu, Limin Han, Yuheng Qiu, Lulin Wang, Mei Wang

**Affiliations:** ^1^ Key Laboratory of Precision Oncology of Shandong Higher Education, Institute of Precision Medicine, Jining Medical University, Jining, China; ^2^ Key Laboratory of Basic Pharmacology of Ministry of Education and Joint International Research Laboratory of Ethnomedicine of Ministry of Education, Zunyi Medical University, Zunyi, China; ^3^ Department of Pathophysiology, Zunyi Medical University, Zunyi, China; ^4^ Key Laboratory of Molecular Pharmacology, Liaocheng People’s Hospital, Liaocheng, China

**Keywords:** miR-365a-3p, gastric cancer, HELLS, aerobic glycolysis, GLUT1

## Abstract

Gastric cancer (GC) is a common and invasive malignancy, which lacks effective treatment and is the third main reason of cancer death. Metabolic reprogramming is one of the main reasons that GC is difficult to treat in various environments. Particularly, abnormal glycolytic activity is the most common way of metabolism reprogramming in cancer cells. Numerous studies have shown that microRNAs play important roles in reprogramming glucose metabolism. Here, we found a microRNA-miR-365a-3p, was significantly downregulated in GC according to bioinformatics analysis. Low expression of miR-365a-3p correlated with poor prognosis of GC patients. Overexpression of miR-365a-3p in GC cells significantly inhibited cell proliferation by inducing cell cycle arrest at G1 phase. Notably, miR-365a-3p induced downregulation of HELLS through binding to its 3′ untranslated region (UTR). Additionally, we found that miR-365a-3p suppressed aerobic glycolysis by inhibiting HELLS/GLUT1 axis. Lastly, we shown that overexpression of miR-365a-3p significantly inhibited tumor growth in nude mice. Conversely, Reconstituted the expression of HELLS rescued the suppressive effects of miR-365a-3p. Our data collectively indicated that miR-365a-3p functioned as a tumor suppressor in GC through downregulating HELLS. Therefore, targeting of the novel miR-365a-3p/HELLS axis could be a potentially effective therapeutic approach for GC.

## Introduction

Gastric cancer (GC) is a common and invasive malignancy, which lacks effective treatment and is the third main reason of cancer death (1, 2). Although the occurrence rate of GC has diminished over past two decades, the mortality remains high. Although some progress has been made in the treatment of GC, including gastrectomy, chemotherapy, radiotherapy and chemotherapy (3), the prognosis of advanced patients remains poor (4, 5). Therefore, there is an urgent need to reveal the underlying mechanisms of gastric carcinogenesis at molecular events, to improve the life quality of GC patients.

Epigenetic changes have been identified that play crucial roles in carcinogenesis, among them, microRNAs (miRNAs) have attracted more attention. MiRNAs are small non-coding endogenous single-stranded RNA, with about 22 nucleotides. The combination of miRNAs with mRNAs for 3′-non-conversion region (UTRs) can induce the formation of miRNA-mRNA complex and lead to the degradation of mRNAs (6, 7). In mammals, miRNAs factor is the key to the regulation of gene expression, to participate in regulation of cell hyperplasia, apoptosis and metabolism, the development of nervous system diseases, cardiovascular disease and cancer (8–10). At present, multiple miRNAs including miR-7, miR-409-3p, miR-221 and miR-155 have been identified as important regulators in GC (11–14). Previous studies have shown that miR-365a-3p is downregulated in some cancers (15–17), but its biological functions in GC are largely unknown.

HELLS (also known as LSH, PASG, and ICF4) is a SNF2-like chromatin-remodeling enzyme, which is transcriptionally regulated by RB/E2F pathway (18, 19). HELLS plays important roles in remodeling chromatin that renders *de novo* DNA methylation and silences gene expression (20, 21). HELLS is low expressed under normal conditions, but it is ubiquitously expressed in proliferating cells such as cancer cells (22). HELLS epigenetically silences multiple tumor suppressor genes and promotes hepatocellular carcinoma progression by regulating chromatin remodeling, such as IGFBP3, E-cadherin, XAF1, FBP1, and CREB3L3 (23). HELLS also can interact with CtIP and to recruits it at the breaks of DNA to promoting DSB repair in cancer cells (24). Down-regulation of HELLS attenuates cell proliferation in glioma and colon cancer (25, 26). HELLS is also required for tumor initiation and progression of retinoblastoma (27). Additionally, HELLS plays important roles in cell metabolism. HELLS interacts with WDR76 to activating glucose metabolism-associated genes, including GLUT1 (28). Moreover, down-regulation of HELLS also reduced glucose consumption and lactate production, demonstrating that HELLS regulates glycolysis (23).

In the study, we detected miR-365a-3p levels in human GC tissues and cells by qRT-PCR, and then investigated function of miR-365a-3p in GC by using gain- or loss of expression approaches for miR-365a-3p. Our data clearly revealed that miR-365a-3p exerted tumor inhibition functions by targeting HELLS, and further suggest that miR-365a-3p-HELLS axis can be a valuable therapeutic target for GC.

## Materials and Methods

### Human Gastric Cancer Tissue Samples

17 human GC tissues and adjacent non-tumor samples were collected from January 2015 to January 2018 at Liaocheng people’s hospital (Liaocheng, China). All samples were frozen in liquid nitrogen, stored at −80°C and used for extraction of RNA. All patients signed the informed consent form. This project was approved by the Institute Research Ethics Committee of Jining Medical University and Liaocheng People’s Hospital. The gene expression omnibus (GEO) database and TCGA used to search for GC-associated miRNA and mRNA expression data sets. Gastric cancer patent clinical information and gene expression data sets were obtained from Oncomir database (http://www.oncomir.org) and KM plotter (http://kmplot.com/).

### Cell Culture

Human GC cell lines MKN-45, HGC-27, SGC-7901 and human normal gastric epithelial RGM-1 cells (Cell Resource Center, Shanghai Institute of Biochemistry and Cell Biology at the Chinese Academy of Sciences, Shanghai, China) were maintained in RPMI 1640 medium containing 10% FBS (Invitrogen), 100 units/ml penicillin (Sigma) and 2 mmol/L l-glutamine at 37 C in a humidified 5% CO2 tissue culture incubator.

### Plasmids, Transfection and Infection

The miR-365a-3p mimics, miR-365a-3p inhibitor and negative controls were obtained from RiBoBio (Guangzhou, China). GC cells were transfected with mimics and inhibitors by using Lipofectamine 3000 (Invitrogen) and collected 48 h after transfection. The plasmid expressing HELLS was obtained from Youbao Biotechnology (Changsha, China). Viral packaging and transduction was performed as precious descrided (29).

### Quantitative Real-Time PCR

The qRT-PCR method has been previously described (29). Briefly, PCR was performed in 96-well plates using three step plus. All reactions performed at five times. Hsa-miR-365a-3p and endogenous control U6 TaqMan microRNA assays were obtained from Applied Biosystems. SYBR Green qRT-PCR was used for qRT-PCR of RNA, and the beta-actin was used to normalize the variation in the cDNA levels. All experiments performed at three times.

### Cell Proliferation Assay

Cell viability was detected using the MTT assay. In brief, the cells were seeded in 96-well plates at a density of 1×10^3^ cells per well and incubated for 1- 5 days. 5 ml of MTT solution (5 mg/ml) was added to each well at different time-points, respectively, and the reactions were subsequently terminated with 200 ml DMSO. Absorbance was measured at 560 nm. All experiments were performed in triplicate.

### BrdU Staining

BrdU staining was performed as previous described (29). BrdU (5-Bromo-2′-Deoxyuridine) was obtained from Sigma. The primary antibody against BrdU (1:200, ab6326, Abcam, Cambridge, USA) and DAPI (300 nM) was used for staining; the percentage of BrdU was calculated.

### Western Blot Analyses

The cells were lysed in RIPA buffer (Beyotime, China). Total protein was separated by 10% SDS-PAGE, and the transferred to a PVDF membrane. The membranes were probed with anti-HELLS, cyclin D1, CDK4, and GLUT1 primary antibodies (Cell Signaling, Danvers, MA) at 4°C overnight, followed by incubation with HRP-conjugated secondary antibody, using GAPDH as the internal control. Proteins were visualized with enhanced chemiluminescence reagents (Pierce, Rockford, IL). Every experiment was repeated at three times.

### Flow Cytometry

For cell cycle analysis, 1 × 10^6^ cells were harvested and washed twice with cold PBS, followed by fixation with ice-cold 70% ethanol overnight at 4°C. After washing twice with PBS, the cells were incubated with propidium iodide (PI) (BD Biosciences, San Jose, CA, USA) and RNaseA for 30 min at room temperature. The cells were then analyzed using a FACS C6 (BD Biosciences, San Jose, CA, USA) with Cell Quest software.

### Luciferase Reporter Assay

For the luciferase assay, MKN-45 and AGS cells were seeded in 96-well plates 24 h before transfection and co-transfected with the HELLS wild-type (Wt) or mutant (Mt) 3′-UTR reporter vector, hU6-miR-365a-3p, or NC and Renilla plasmid using Lipofectamine 2000 (Invitrogen). Luciferase activities were determined with the Dual-Luciferase Reporter System (Promega) according to the manufacturer’s instructions.

### Glucose Uptake and Consumption Assays

For glucose uptake assay, 2000 cells were seeded in 96-well plates with glucose-free medium overnight, wash cell three times in PBS. Starve cells for glucose by pre-incubating with 100 µl KRPH buffer for 10 minutes. Added 2-DG to cells and incubate for 20 min at 37°C. 2-DG6P levels were determined with microplate reader in kinetic mode at 37°C according to the manufacturer’s instructions (Abcam ab136955). For glucose consumption assay, 2×10^5^ cells were seeded in plates at 37°C for 48 h, the glucose content was detected by using a Glucose Assay kit (Sigma GAGO20). Data were analyzed according to standard curve line and OD value. All experiments were performed at three times.

### Lactate and Lactate Dehydrogenase (LDH) Assays

The lactate and LDH assays were performed according to the manufacturer’s instructions (Sigma MAK064 and MAK066). In brief, 2 × 10^5^ cells were seeded in plates at 37°C for 48 h. Samples were treated as manufacturer’s instructions, OD value was analyzed by using a SYNERGY HTX multi-mode reader. All experiments were performed in triplicate.

### Extracellular Acidification Rate (ECAR) Assay

Seahorse XF-96p analyzer was used to detect real-time status changed of ECAR. GC cells with miR-365a-3p mimics or NC were seeded into XF96 cell culture microplates at 40000 cells/well and cultured for 24 h. Then replaced medium with Seahorse DMEM containing 2 µM glutamine, and the microplates were maintained in a non-CO2 incubator at 37°C for 60 min. The data were analyzed to cell numbers and plotted as ECAR (mpH/min) as a function of time.

### Tumor Xenograft Experiment

Animal studies were carried out as previous described (30), in briefly; female SCID mice (5 weeks old) were purchased and housed in an SPF room. GC cells (1 × 10^6^) were injected subcutaneously into the flanks of nude mice following a previous protocol with minor modifications (30). For intratumoral injection of cholesterol-conjugated RNA, miR-Ribo agomir-365a-3p, 2 nmol RNA in 50 µl saline buffer was locally injected into each tumor mass at a 3-day interval for 24 days. The tumor size was measured using a vernier caliper every 5 days. Lastly, the tumor mass was harvested, weighed, and stored for immunostaining. All studies were approved by the Animal Care and Use Committee of Jining medical university. Animal welfare and experimental procedures were carried out in accordance with the *Guide for the Care and Use of Laboratory Animals* (Ministry of Science and Technology of China, 2006).

### Immunohistochemical Staining

Immunohistochemical staining was carried as previous described (31). The antibodies HELLS (1:500; Santa Cruz, sc-46665) and GLUT1 (1:250; Abcam, ab115730) were used in this study.

### Statistical Analysis

All experiments were repeated at least three independent experiments. Data were collected and analyzed using Graphpad Prism 7. Two-tailed Student’s t-test was performed for paired samples. Quantitative data are expressed as the mean ± standard deviation. P < 0.05 was considered statistically significant.

## Results

### MiR-365a-3p Was Low Expressed in GC and Low Expression of miR-365a-3p Correlates With Poor Patient Prognosis

Initially, GEO data GSE54397 and TCGA GC patients’ miRNA data were downloaded and analyzed. 34 down-regulated miRNAs were respectively obtained from GC samples and normal samples in GSE54397 data set (**Figure 1A**). We further explored GC-related miRNAs between 20 top down-regulated miRNAs in GSE54397 and 30 top down-regulated miRNAs in TCGA data sets by using Venn analysis. Here, miR-486-5p and miR-365a-3p were found in the intersection of the two data sets (**Figure 1B**). Previous studies have identified that miR-486-5p functioned as a tumor suppressor in GC (32). Therefore, we focused on miR-365a-3p in this study. We detected the expression of miR-365a-3p in fresh GC and normal tissues. In line with TCGA data, miR-365a-3p was also abnormally attenuated in fresh GC compared with the adjacent tissues (**Figure 1C**). In addition, miR-365a-3p significantly correlated with probability of survival and patients with low level of miR-365a-3p had a poor prognosis (**Figure 1D**). Consistently, compared to normal gastric RGM-1 cells, miR-365a-3p was also significantly decreased in GC cell lines (**Figure 1E**).

**Figure 1:** MiR-365a-3p was downregulated in GC and low expression of miR-365a-3p correlates with poor patient prognosis. **(A)** Heatmap showing down-regulated miRNAs in GSE54397 data set. **(B)** The intersection of differentially expressed miRNAs in GC-related expression data sets. The left circle is the top 20 down-regulated miRNAs in the GSE54397 expression data set. The right circle is top 30 down-regulated miRNAs in TCGA data sets. **(C)** The expression of miR-365a-3p in the TCGA expression data set and local cohort. **(D)** Kaplan–Meier analysis of overall survival from the Oncomir database with the log rank test *P* value indicated. **(E)** qRT-PCR analysis of miR-365a-3p expression in RGM-1, HGC-27, SGC7901, AGS and MKN-45 cells. All data were shown as the mean ± SD, *p < 0.05, **p < 0.01. All p values were based on analysis control versus treatment.

### MiR-365a-3p Inhibited GC Cell Proliferation

To explore the effect of miR-365a-3p in ability of cell proliferation, miR-365a-3p was over-expressed in GC cells *via* transfection and MTT assay was performed. As shown, overexpression of miR-365a-3p evidently repressed proliferation compared to control group (**Figures 2A, B**). On the contrary, the proliferation of GC cells was significantly increased after transfection with antisense miR-365a-3p (**Figures 2C, D**). The above result was confirmed by BrdU incorporation test in GC cells. Our data showed that DNA synthesis of miR-365a-3p over expression cells diminished about 40%, and miR-365a-3p knockdown cells raised by more than 60% in DNA synthesis compared to control cells (**Figures 2E, F**). These data clearly suggested that miR-365a-3p repressed cell proliferation in GC.

**Figure 2:** MiR-365a-3p suppressed cell proliferation in GC. **(A, B)** MKN-45 and AGS cells transfected with miR-365a-3p-expressing or control mimics. The expression of miR-365a-3p was detected by qRT-PCR analysis **(A)** and cell proliferation was examined by MTT assays **(B)**. **(C, D)** MKN-45 and AGS cells transfection with miR-365a-3p-expressing or control inhibitor. The expression of miR-365a-3p was detected by qRT-PCR analysis **(C)** and cell proliferation was examined by MTT assays **(D)**. **(E, F)** Image and quantification of MKN-45 and AGS cells positive for BrdU staining. All data were shown as the mean ± SD, *p < 0.05, **p < 0.01.

### MiR-365a-3p Induced Cell Cycle Arrest in GC

We analyzed cell cycle progression to determine whether miR-365a-3p represses cell proliferation through blocking cell cycle process. Indeed, after miR-365a-3p mimics treatment, the amount of cells was accumulated in G1 phase (**Figures 3A, B**). Inversely, inhibition of miR-365a-3p triggered cell cycle progression in GC (**Figures 3C, D**). Further studies showed that the expression of CDK4 and cyclin D1 was decreased after miR-365a-3p overexpression, while inhibition of miR-365a-3p promoted the levels of cyclin D1 and CDK4 (**Figure 3E**). Immunoblotting quantifications were shown in **Figure 3F**. These results further indicated that miR-365a-3p-mediated cell proliferation inhibition was linked to cell cycle arrest at G1 phase.

**Figure 3:** MiR-365a-3p suppressed the cell cycle progression of GC cells by inhibiting cyclin D1 and CDK4. After miR-365a-3p mimics **(A)** or inhibitor **(B)** were transfected, the distribution of cell cycle was detected by flow cytometry. **(C, D)** The experiments were repeated 3 times with similar results and representative graphs were illustrated. **(E)** Expression of cyclin D1 and CDK4 were examined by western blot. **(F)** Quantitative analysis of cyclin D1 and CDK4 expression in miR-365a-3p-modulated cells. All data were shown as the mean ± SD, *p < 0.05, **p < 0.01.

### HELLS Was a Direct Target of miR-365a-3p

To further understanding the tumor inhibitory mechanism of miR-365a-3p in GC, top 300 high expressed mRNAs of TCGA data were employed. In order to find the potential targets of miR-365a-3p in GC, we used two independent online database miRanda and TargetScan. The predicted genes were intersected with the top 300 up-regulated genes in TCGA data set by using Venn analysis. HELLS was identified in the intersection of three data sets, which plays important roles in cancer development and progression (**Figure 4A**). Next, we predicted the seed region-binding site of miR-365a-3p on HELLS 3′-UTR by using TargetScan (**Figure 4B**). On this basis, we then constructed the HELLS 3′ UTR reporting system and detected whether HELLS was a target of miR-365a-3p by luciferase analysis. We found that miR-365a-3p profoundly diminished the luciferase activity of HELLS plasmid-transfected cells containing wild-genre 3′ UTR. While cells were transfected with HELLS mutant-genre 3′ UTR plasmid, the luciferase activity was unchanged (**Figure 4C**). In addition, compared to normal gastric cells GES-1, the expression of HELLS was increased in GC cells (**Figure 4D**). Furthermore, miR-365a-3p mimic or antagomir were transfected in to GC cells and HELLS expression was detected by WB and qRT-PCR assay. Overexpression of miR-365a-3p reduced HELLS expression. In contrast, inhibition of miR-365a-3p increased HELLS expression in gastric cancer cells (**Figures 4E, F**). Quantitative RT-PCR analysis further confirmed these results (**Figure 4G**). In conclusion, above results suggested that miR-365a-3p directly inhibited HELLS through binding its 3′ UTR region.

**Figure 4:** MiR-365a-3p directly targeted the HELLS 3′-UTR. **(A)** The intersection of miR-365a-3p targeting gene prediction and up-regulated gene in the TCGA data set. HELLS was identified in the intersection of three data sets. **(B)** Wild-type and mutant miR-365a-3p target sequences of the HELLS 3′-UTR. **(C)** Relative luciferase activity of MKN-45 and AGS cells after co-transfection with wild-type (Wt) or mutant (Mt) HELLS 3′-UTR reporter genes along with miR-365a-3p or NC. **(D)** Western blot analysis to determine the expression of HELLS in immortalized human gastric mucosal epithelial cell line and GC cell lines. **(E, F)** western blot and **(G)** qRT-PCR analysis of HELLS expression in GC cells transfected with miR-365a-3p mimics or inhibitors. All data are shown as the mean ± SD, **p < 0.01.

### MiR-365a-3p Attenuated Aerobic Glycolysis of GC Cells *via* Regulating HELLS

To further exploring the function of miR-365a-3p in biological process, we focused on whether miR-365a-3p regulates aerobic glycolysis in GC cells. We found that overexpression of miR-365a-3p remarkably decreased glucose uptake of GC cells (**Figure 5A**). GO assay showed that miR-365a-3p overexpression significantly inhibited glucose consumption of GC cells (**Figure 5B**). In addition, lactate production as well as LDH activities were significantly attenuated in miR-365a-3p-overexpressed cells, compared with control cells (**Figures 5C, D**). Then, we performed glycolytic stress flux test to detect the changes of glycolytic flux by using Seahorse XF-96p analyzer. The results demonstrated that glycolytic flux was attenuated after miR-365a-3p overexpression in GC cells (**Figure 5E**). Moreover, ATP assays showed that overexpression of miR-365a-3p increased the inhibition rate of ATP induced by oligomycin (**Figure 5F**). Next, we detected the expressions of key glycolysis-associated enzymes in miR-365a-3p overexpression cells. We found that miR-365a-3p regulated glycolysis by modulating GLUT1 expression, but not GLUT4, FBP1, HK2, and PKM2 levels (**Supplemental Figure S1**). All these results suggested that miR-365a-3p attenuated aerobic glycolysis in GC cells.

**Figure 5:** MiR-365a-3p inhibited aerobic glycolysis by regulating HELLS-GLUT1 axis. **(A)** Glucose uptake of MKN-45 and AGS cells transfected with miR-365a-3p-expressing or control mimics. **(B)** Glucose consumption of MKN-45 and AGS cells transfected with miR-365a-3p-expressing or control mimics. **(C)** Lactate production of MKN-45 and AGS cells transfected with miR-365a-3p-expressing or control mimics. **(D)** Lactate dehydrogenase activities of MKN-45 and AGS cells transfected with miR-365a-3p-expressing or control mimics. **(E)** Glycolytic flux changes of MKN-45 and AGS cells transfected with miR-365a-3p-expressing or control mimics. ECAR, extracellular acidification rate. **(F)** ATP inhibition induced by oligomycin in GC cells with or without miR-365a-3p overexpression. **(G, H)** Immunoblotting of HELLS and GLUT1 in MKN-45 and AGS cells transfected with miR-365a-3p-expressing mimics with or without HELLS restoration. **(I)** Glucose uptake of MKN-45 and AGS cells transfected with miR-365a-3p-expressing mimics with or without HELLS restoration. **(J)** Glucose consumption of MKN-45 and AGS cells transfected with miR-365a-3p-expressing mimics with or without HELLS restoration. **(K)** Lactate production of MKN-45 and AGS cells transfected with miR-365a-3p-expressing mimics with or without HELLS restoration. All data were shown as the mean ± SD, *p < 0.05, **p < 0.01.

Some studies have demonstrated that HELLS could regulate glycolysis (23, 28). Our results showed that knockdown of HELLS significantly suppressed glucose uptake and glycolysis, which was recused by the reconstituted expression of HELLS (**Supplemental Figure S2**). To further evaluating whether miR-365a-3p inhibits glycolysis by regulating HELLS, we restored HELLS expression in miR-365a-3p-overexpressed GC cells. We found that the expression of well-known glycolytic gene GLUT1, which was targeted by HELLS, was significantly up-regulated after HELLS restoration (**Figures 5G, H**). Besides this, glucose uptake, glucose consumption and lactate production were also increased when HELLS re-overexpression after miR-365a-3p overexpression (**Figures 5I–K**). These results showed that miR-365a-3p affected aerobic glycolysis by directly inhibiting HELLS.

### MiR-365a-3p Suppresses Tumorigenesis by Regulating HELLS-GLUT1 Axis in GC

Since HELLS was a direct target of miR-365a-3p in GC, we next detected clinical significance of HELLS in GC patients. The TCGA mRNAs data was used to evaluate the expression of HELLS in GC, the results showed that HELLS was significantly up-regulated in GC than normal tissues (**Figure 6A**). The results of our local cohort also showed that the expression of HELLS was higher in GC than that in adjacent non-tumor samples, which further confirmed TCGA results (**Figure 6B**). The survival data from TCGA was used to explore the effects of HELLS on overall survival. We found that high expression of HELLS was correlated with reduced survival time of GC patients (**Figure 6C**). In addition, we evaluated the correlation of miR-365a-3p and HELLS expression in GC patients, the results showed that HELLS was negatively correlated with miR-365a-3p in our local specimens (**Figure 6D**).

**Figure 6:** MiR-365a-3p-HELLS axis regulated GC progression. **(A, B)** Box plot of HELLS expression levels from gastric normal tissues and GC tissues in TCGA data set and our local cohort data. **(C)** Kaplan–Meier analysis of overall survival for the KM plotter database with the log rank test *P* value. **(D)** The inverse correlation between miR-365a-3p and HELLS in local patient cohort. **(E)** Representative tumor tissues extracted from mice inoculated with MKN-45 cells expressing miR-365a-3p or NC. **(F)** Measurement of tumor volumes at the indicated time-points. **(G)** Immunohistochemistry of HELLS and GLUT1 in indicated tumor tissues. All data are shown as the mean ± SD, **p < 0.01. All p values are based on analysis control versus treatment.

To further detect the effect of miR-365a-3p and HELLS on tumor formation *in vivo*, we injected MKN-45/vector and MKN-45/HELLS cells subcutaneously into SCID mice to observe tumor growth. MiR-Ribo agomir-365a-3p and NC were locally injected into each tumor mass at a 3-day interval for 24 days. These results revealed that upregulation of miR-365a-3p repressed tumor formation of GC cells. In addition, the averages of tumor weight and volume of miR-365a-3p overexpression group were lower than those in negative controls (NC), which was rescued by the HELLS overexpression (**Figures 6E, F**). Besides, the expression of GLUT1 in miR-365a-3p-overexpression tumors was decreased compared with controls, whereas this effect was recovered by restored expression of HELLS (**Figure 6G**). These results further indicated that miR-365a-3p suppresses tumor growth *via* the HELLS-GLUT1 axis mediated aerobic glycolysis in GC.

## Discussion

The prognosis of patients with gastric cancer remains poor, partly due to resistance to treatment. Therefore, it is very crucial to further understanding the molecular pathogenesis of GC development, and to improve the live quality of GC patients. Previous studies have identified that some representative miRNAs were differentially expressed in GC. In the study, we found that miR-365a-3p might play an anti-tumor role in GC by targeting HELLS.

MiR-365a-3p is located at 16p13.12, which is involved in cancer development. We found that expression of miR-365a-3p was evidently decreased in GC, suggesting its tumor suppressive functions. Previous studies have demonstrated that miR-365a-3p inhibited proliferation and metastasis in lung cancer cells (16). Similar roles are found in pancreatic cancer and other cancers (33, 34). We found that miR-365a-3p repressed proliferation by inducing cell cycle arrest at G1 phase in GC. Reversely, inhibition of miR-365a-3p promoted cell proliferation. Additionally, cyclin D1 and CDK4, which promote the continuity from G1 to S phase, were also regulated by miR-365a-3p. These data suggested that miR-365a-3p inhibited cell proliferation by suppressing cell cycle progression, and overexpression of miR-365a-3p inhibited tumor formation, which further support the conclusion that miR-365a-3p plays an anti-cancer role in GC.

HELLS (also known as LSH, PASG and ICF4) is a SNF2-like chromatin remodeling enzyme, which regulates cell hyperplasia, differentiation and apoptosis by activating complex signal cascades (35–38). In this study, we used two separate bioinformatics databases to predict that miRNAs could be combined with HELLS mRNA’s 3′ UTR. In these miRNAs, miR-365a-3p is clearly identified in two databases. Our data identified that HELLS was a direct target of miR-365a-3p. Firstly, miR-365a-3p significantly inhibited activity of HELLS 3′-UTR luciferase reporter, but the mutation of “seed region” abolished this impact. Secondly, overexpression of miR-365a-3p decreased HELLS expression.

Some studies have demonstrated that HELLS played important roles in glycolysis, that could activate the transcription of GLUT1 (23, 28). Here, we demonstrated that miR-365a-3p attenuated aerobic glycolysis by decreasing the expression of GLUT1 in GC cells. In addition, reintroduction of HELLS could abrogate the effects induced by miR-365a-3p overexpression. Based on these results, we suggest that miR-365a-3p represses GC cell glycolysis, proliferation and tumor formation, partly by inhibiting HELLS. As to the outcomes, some recent studies showed that low miR-365a-3p correlated with poorer survival time (16, 33, 34). On the contrary, there are several evidences that high HELLS expression correlated with poorer prognosis (23, 39, 40). The contrary impact of miR-365a-3p and HELLS in cancer outcomes provides an in immediate evidence to support the anti-cancer function of miR-365a-3p in GC.

Taken together, miR-365a-3p is significantly downregulated in GC. MiR-365a-3p represses cell aerobic glycolysis, proliferation and tumor formation by targeting HELLS-GLUT1 axis, in which miR-365a-3p negatively regulates HELLS by binding to 3′ UTR of HELLS mRNA in GC cells. Our data indicate that targeting miR-365a-3p-HELLS axis will have clinical and translational significance.

## Data Availability Statement

The original contributions presented in the study are included in the article/**Supplementary Material**. Further inquiries can be directed to the corresponding authors.

## Ethics Statement

The studies involving human participants were reviewed and approved by the ethics committee of Liaocheng People’s Hospital. The patients/participants provided their written informed consent to participate in this study. The animal study was reviewed and approved by Institute for Laboratory Animal Research, Jining Medical University.

## Author Contributions

Conception and design: RY and MW. Acquisition of data: RY, GL, LH, LW, and YQ. Analysis and interpretation: RY, GL, and MW. Original manuscript drafting and figure construction: RY. Manuscript editing and completion: RY and MW. All authors contributed to the article and approved the submitted version.

## Funding

This work was supported by the National Natural Science Foundation of china (no. 82002639 to RY), Shandong Provincial Natural Science Foundation, China (No. ZR2020QH235 to RY) and faculty start-up fund for RY from Jining Medical University.

## Conflict of Interest

The authors declare that the research was conducted in the absence of any commercial or financial relationships that could be construed as a potential conflict of interest.
